The article "MicroRNA-10a Is Down-Regulated by DNA Methylation and Functions as a Tumor Suppressor in Gastric Cancer Cells" was retracted in 2023. Reasons: compromised peer review; concerns about the images; concerns about the authorship.

# MicroRNA-10a Is Down-Regulated by DNA Methylation and Functions as a Tumor Suppressor in Gastric Cancer Cells

**DOI:** 10.1371/journal.pone.0088057

**Published:** 2014-01-31

**Authors:** Hongyan Jia, Zhengyi Zhang, Dongling Zou, Bin Wang, Yunmeng Yan, Min Luo, Lei Dong, Haixin Yin, Bei Gong, Zheng Li, Fang Wang, Wei Song, Changzheng Liu, Yanni Ma, Junwu Zhang, Haoliang Zhao, Jianxiong Li, Jia Yu

**Affiliations:** 1 Department of Biochemistry, Institute of Basic Medical Sciences, Chinese Academy of Medical Sciences (CAMS) & Peking Union Medical College (PUMC), Beijing, PR China; 2 Cancer center, The General Hospital of the People's Liberation Army, Beijing, PR China; 3 Department of Surgery, The First Hospital of Shanxi Medical University, Taiyuan, PR China; 4 Department of Gynecologic Oncology, Chongqing Cancer Institute, Chongqing, PR China; 5 Department of Surgery,The Shanxi Academy of Medical Sciences & Shanxi Dayi Hospital, Taiyuan, PR China; CEA - Institut de Genomique, France

## Abstract

**Background:**

MicroRNAs act as posttranscriptional regulators of gene expression in many biological processes. Their deregulations occur commonly in gastric cancer (GC). Although DNA methylation constitutes an important mechanism for microRNA deregulation in cancer, this field largely remains unexplored.

**Methodology/Principal Findings:**

Total RNA was extracted from the tissues of 100 patients with GC and four gastric cancer cell lines. The expression levels of miR-10a were determined by real-time PCR with specific TaqMan probes. Moreover, a functional analysis of miR-10a in regulating cell proliferation, migration and invasion was performed. Subsequently, quantitative methylation-specific PCR (qMSP) was used to detect the DNA methylation status in the CpG islands upstream of *miR-10a*. In this study, we found that the expression of miR-10a in GC cells was lower than that in normal cells, which was due to the hypermethylation of the CpG islands upstream of *miR-10a*. We also validated the slightly lower expression of miR-10a in GC tissues than their adjacent non-neoplastic tissues in 100 GC patients and confirmed the hypermethylation of CpG islands upstream of *miR-10a* in some patients. Furthermore, re-introduction of miR-10a into GC cells was able to inhibit cell proliferation, migration and invasion. Bioinformatic and immunoblot analysis indicated that the tumor suppressor roles of miR-10a in GC cells were possibly through targeting HOXA1.

**Conclusions/Significance:**

Our data indicate that miR-10a acts as a tumor suppressor in GC cells and is partially silenced by DNA hypermethylation in GC, suggesting that miR-10a may serve as a potential diagnostic or therapeutic target of GC.

## Introduction

Gastric cancer (GC) is the second most frequent cause of death from cancer in the world [1]. Thus far, few tumor suppressor genes and tumor-related genes have been reported in GC. Although extensive studies have been performed to identify genetic pathways and mechanisms involved in cancer development, few improvements on the early diagnosis of cancer have been made. MicroRNAs (miRNAs) are endogenous small non-coding RNAs that have been identified as posttranscriptional regulators of gene expression. Previous studies have indicated that miRNAs exert their functions through imperfect base-pairing with the 3′untranslated region (3′UTR) of target mRNAs [2] and miRNAs have been extensively studied in the context of cell cycle regulation, differentiation, development and apoptosis [3], [4]. Accumulated evidence indicates that miRNAs are deregulated in various diseases, especially in cancer. For example, miR-216b is markedly down-regulated in nasopharyngeal carcinoma [4]; miR-340 is deregulated in breast cancer and can inhibit breast cancer cell migration and invasion [5]; and miR-31 was identified as an oncogene in esophageal squamous cell carcinoma [6]. Taken together, miRNAs have been identified as potential candidates for novel diagnostic biomarkers or therapeutic targets of cancer.

MiR-10a has been reported to play important roles in the genesis and development of a variety of human cancers. For example, miR-10a is deregulated in head and neck squamous cell carcinomas and also in hepatocellular carcinoma [7], [8]. Furthermore, in human cervical cancer, miR-10a serves as an oncogene by regulating CHL1 [9]; down-regulation of miR-10a in chronic myeloid leukemia promotes CD34^+^ cells proliferation [10]. However, the function of miR-10a and the mechanism underlying gastric carcinogenesis remain unclear. In this study, we accurately measured the expression of miR-10a in 100 patients with gastric cancer and investigated the roles of miR-10a in gastric cancer cells. We found that miR-10a was down-regulated in GC tissues and enforced expression of miR-10a repressed the proliferation, migration and invasion of GC cells.

Epigenetic modifications including DNA hypermethylation, histone deacetylation and histone methylation are closely associated with gene inactivation. Promoter hypermethylation is thought to be an alternative mechanism to down-regulate tumor suppressor genes in human cancers [11]. MiRNAs whose expression is repressed by DNA methylation have been reported in a few human cancers [12]–[14]. To further investigate whether the down-regulation of miR-10a originates from the hypermethylation of the genomic region upstream of *miR-10a*, we analyzed the DNA methylation of CpG island in the promoter region of *miR-10a* in 55 GC patients and found that down-regulation of miR-10a in GC tissues might be due to the hypermethylation of CpG sequences in its promoter.

## Materials and Methods

### Patients and Specimens

Human clinical samples were collected from surgical specimens from 100 patients with GC at Cancer Institute and Hospital, Chinese Academy of Medical Sciences, General Hospital of the People's Liberation Army and Shanxi Cancer Hospital. The corresponding adjacent non-neoplastic tissues from the macroscopic tumor margin were isolated at the same time and used as controls. Tumors were staged according to the TNM (2010) classification criteria of the Union for International Cancer Control (UICC). All samples were divided into two parts and were immediately snap frozen in liquid nitrogen and stored at −80°C until RNA extraction. Four gastric cancer cell lines (HGC-27, MGC-803, SGC-7901 and MKN-45) were all preserved in our laboratory and maintained in DMEM or 1640 with 10% FBS. The Clinical Research Ethics Committee of Institute of Basic Medical Sciences, Chinese Academy of Medical Sciences approved the research protocols and written informed consent was obtained from the participants.

### RNA Extraction, cDNA Synthesis of mRNAs and miRNAs, and Real-time PCR Assays

Total RNA was extracted from gastric cancer tissues and cells using Trizol reagent (Invitrogen, CA, USA) according to the manufacturer’s instructions. RNA was quantified by absorbance at 260 nm and cDNA was synthesized by M-MLV reverse transcriptase (Invitrogen) from 2 µg of total RNA. Oligo (dT) 18 was used as the RT primers for reverse transcription of mRNA. A stem-loop RT primer was used for the reverse transcription of miRNA. Quantitative RT-PCR was performed in a Bio-Rad CFX96 real-time PCR System (Bio-Rad, CA, USA) using SYBR Premix Ex Taq kit (Takara, Dalian, China) or TaqMan probes (Applied Biosystems, Foster City, CA, USA) according to the manufacturer’ s instructions. The PCR conditions were as follows: 95°C for 30 s, followed by 40 cycles of 95°C for 5 s and 60°C for 34 s. For mRNAs, the data were normalized using the endogenous GAPDH control. For miRNAs, U6 snRNA was used as the endogenous control. The relative amount of miR-10a was measured with the 2^−ΔΔCT^ method. Primer sequences are presented in Table S1.

### DNA Extraction, Methylation-specific PCR (MSP) and Quantitative Methylation-specific PCR (qMSP)

High molecular weight genomic DNA was extracted from gastric cancer tissues using a DNA Extraction Kit (biomed, BJ, China) according to the manufacturer’s instructions. Bisulfite modification was performed using the Epitect Bisulfite sequencing kit (Qiagen, Hilden, Germany) according to the protocol. Up to 2 µg of genomic DNA was used as a starting material. Normal lymphocyte DNA treated with CpG Methyltransferase (M.SssI) (NEB, MA, USA) was used as a positive control, and a reaction system without any template was used as a blank control.

The sodium bisulfate-treated DNA was amplified using the Bio-Rad CFX96 real-time PCR System (Bio-Rad) using KAPA SYBR® FAST qPCR Kits (Kapa Biosystems) with the following conditions: 95°C for 5 min followed by 40 cycles of 95°C for 30 s, 54°C for 30 s and 72°C for 30 s and a final extension at 72°C for 10 min. GAPDH was used as an internal control. qMSP reactions were performed in triplicate. The methylation level in a sample was estimated as Lu L et al. described [15]. Primer sequences are presented in Table S1.

### 5-Aza-2′-deoxyazacytidine Treatment

Gastric cancer cells were seeded in 10 cm dishes (1×10^6^ cells per dish) one day before drug treatment. The cells were treated with 1 µM 5-Aza-2**′**-deoxyazacytidine (5-AZA) (Sigma, MO, USA) every 24 h for 3 days.

### Cell Culture and Oligonucleotides Transfection

The human gastric cell lines HGC-27, SGC-7901 and MKN-45 were cultured in RPMI 1640 (Gibco, BRL, UK) media supplemented with 10% fetal bovine serum, and MGC-803 was maintained in DMEM (Gibco, BRL, UK) supplemented with 10% fetal bovine serum. These cell lines were maintained at 37°C in humidified air containing 5% CO_2_.

The miR-10a mimic, the scramble mimic, siHOXA1 siRNA and scramble siRNA were synthesized by GenePharma (Shanghai, China) and transfected into the cells at a final concentration of 50 nmol/L using DharmaFECT1 Reagent (Dharmacon, TX, USA).

### Cell Proliferation and Colony Formation Assay

The mimic- or siRNA- transfected cells were seeded into 96-well plates (5000 cells/well). Cells were incubated with 10% CCK-8 (DOJINDO, Japan) at 37°C until visual color conversion occurred. Proliferation rates were determined at 0, 12, 24, 48, 72, 96 hours after transfection.

The mimic-transfected cells were trypsinized and replated at 200 cells per well in 6-well plates and maintained in 1640 with 10% FBS. The cells were cultured for 7 days, fixed with methanol and stained with 0.1% crystal violet in 20% methanol for 15 min.

### Cell Apoptosis Assay

Apoptosis assays were performed in HGC-27 and MGC-803 cell lines using the Annexin V-FITC Apoptosis Detection kit I (BD Biosciences) according to the manufacturer's protocol and then analyzed by Calibur Flow Cytometer (BECTON DICKINSON).

### Cell Migration and Invasion Assays

A wound-healing assay was performed to assess cell migration. An artificial wound was created on a confluent cell monolayer without FBS using a 200 µL pipette tip 24 hours after transfection. To visualize migrating cells and wound healing, images were taken at 0, 12, 24, 36, 48, 60 hours.

For the transwell invasion assays, HGC-27 and MGC-803 cells suspended in 0.2 ml RPMI 1640 or DMEM without FBS were placed on the top chamber of each insert (Millipore, MA, USA) precoated with 40 µl of 1 mg/ml matrigel. The lower chamber was filled with 600 µl of RPMI 1640 or DMEM medium with 10% FBS as the nutritional attractant. 24 hours later, the invasion cells attached to the lower surface were fixed with 20% methanol and stained with May-Gruwald-Giemsa (MGG). The membranes were then carved and embedded under cover slips. Cells in three different visual fields were counted, and all assays were performed in triplicate.

### Western Blotting

Western blot analysis was performed according to standard methods. Proteins were separated by 10% SDS-PAGE and then transferred to PVDF membranes (Amersham, Buckinghamshire, UK). Membranes were blocked overnight with 5% non-fat dried milk and incubated for 2 h with an anti-HOXA1 antibody (Bioworld, MN, USA) at 1∶500 dilutions or anti-GAPDH antibody (Proteintech, Chicago, USA) at 1∶50,000 dilutions. After washing with TBST (10 mM Tris, pH 8.0, 150 mM NaCl, and 0.1% Tween20), the membranes were incubated for 2 h with secondary antibody (zsgb-bio, Beijing, China).

### Statistics

Each experiment was repeated at least three times. The student's t test (two-tailed) and the x^2^ test were performed, and statistical significance was defined as α = 0.05 (two-side). The means ± SD are displayed in the figures.

## Results

### miR-10a is Down-regulated in Gastric Cancer Cells

We examined the expression of mature miR-10a in four human gastric cancer cell lines (HGC-27, MGC-803, SGC-7901 and MKN-45) and a human gastric epithelium cell line (GES). The expression level of miR-10a in GES was significant higher than the levels in the two gastric cancer cell lines (HGC-27 and MGC-803) and was non-significantly but observably higher than the levels in the other two gastric cancer cell lines (MKN-45 and SGC-7901) (FIG. 1a). These data suggested that the down-regulation of miR-10a might be relevant to the genesis and development of GC.

**Figure 1:** The expression of miR-10a in human gastric cancer cell lines and clinical GC samples. **a** The expression of miR-10a in four human gastric cancer cell lines (HGC-27, MGC-803, SGC-7901 and MKN-45) and a human gastric epithelium cell line (GES) was detected using real-time PCR with TaqMan probes. **b** The expression of miR-10a in 100 pairs of GC tissues compared with their matched adjacent non-neoplastic tissues. **c** The expression of miR-10a in the GC tissues was lower than that in adjacent tissues, although there were no statistically significant differences. P = 0.148, paired t-test, two-tailed. U6 snRNA was used as the endogenous control.

### The Expression of miR-10a in Clinical GC Patients and their Correlation with Clinicopathological Characteristics

To further study the relationship between miR-10a and GC genesis, we detected the expression of miR-10a in 100 clinical patients by TaqMan probe-derived real-time PCR as described above. Out of 100 pairs of GC samples, the expression of miR-10a was down-regulated in 58 cases (58/100, 58%) compared with the corresponding adjacent tissues (FIG. 1b). Overall, the expression of miR-10a was down-regulated in GC tissues compared with the adjacent tissues, although the down-regulation was not statistically significant (p = 0.148, paired t-test, two-tailed) (FIG. 1c).

To evaluate the correlation between the expression of miR-10a and the clinicopathological characteristics, the patients were divided into two groups according to the relative expression of miR-10a in cancer tissues according to a previously published paper [16]. As shown in Table S2, a statistically significant association was observed between the two TNM groups. There are more patients who are in I+II stage in the group with lower expression of miR-10a in their GC tissues. This relationship indicated that miR-10a may be more important in early cancer carcinogenesis. However, our data demonstrated that the expression level of miR-10a had no correlation with age, gender, histological type, tumor percentage, venous invasion, nerve invasion, position, Borrmann typing, pT stage, pN stage or pM stage.

### miR-10a Inhibits Cell Proliferation *in vitro*

To explore the role of miR-10a in gastric carcinogenesis, we transfected miR-10a mimic into the GC cell lines HGC-27 and MGC-803, both of which exhibited high transfection efficiency (FIG. 2a). As demonstrated by CCK-8 growth assays 0, 1, 2, 3 and 4 days after mimic transfection, overexpression of miR-10a reduced cell proliferation in both cell lines, whereas the scramble mimic had no effect on cell proliferation compared with the untreated cells (FIG. 2b). Subsequently, colony formation assays were performed to evaluate the proliferative ability of mimic-transfected HGC-27 and MGC-803 cells and revealed that overexpression of miR-10a in HGC-27 cells reduced colony formation (FIG. 2c). However, none of the MGC-803 cells formed colonies, which might be due to the cells’ relatively weak adherence. To further address the effect of miR-10a on cell apoptosis in the two GC cell lines, the early apoptosis of MGC-803 and HGC-27 cells was examined by Annexin V staining after miR-10a mimic transfection. As expected, few early apoptotic cells (20.8% in HGC-27 and 22.9% in MGC-803) were detected in the scramble mimic-treated cells, whereas miR-10a mimics treatment increased the percentage of early apoptotic cells (28.4% in HGC-27 and 27.7% in MGC-803) (FIG. 2d). Collectively, we concluded that miR-10a could suppress cell survival in GC cells by inducing cell apoptosis.

**Figure 2:** miR-10a inhibits cell proliferation *in vitro*. **a** miR-10a expression in HGC-27 and MGC-803 cells transfected with 50 nmol/L scramble or miR-10a mimic for 48 h. **b** Growth assays by cck-8 at 0, 1, 2, 3, 4 days after mimic transfection. **c** Colony formation assay of untreated, scramble-transfected, and miR-10a-transfected HGC-27 cells. **d** MGC-803 and HGC-27 cells were stained with PE Annexin V and 7-AAD 72 h after treatment with miR-10a mimics or scramble. Early apoptotic cells are shown in the bottom right quadrant. All data are presented as the means ± SD. *, P<0.05; **, P<0.01, ***, P<0.001.

### miR-10a Inhibits Cell Migration and Invasion *in vitro*

We further assessed the effects of miR-10a on cell migration and invasion, which were the key determinants of malignant progression and metastasis. The migration ability was demonstrated by a wound healing/scratch assay in HGC-27 and MGC-803 cells. Both of cell lines treated with miR-10a mimic were distinctively less migratory than those treated with the scramble control or untreated cells at 12, 24, and 36 hours after scratching (FIG. 3a). Furthermore, we conducted a Matrigel cell invasion assay and stained the invaded cells to measure the directional invasion abilities of the cells after ectopically expressing miR-10a in the two cell lines. The invasiveness of cells transfected with miR-10a mimic was dramatically decreased compared with the scramble control and untreated cells (FIG. 3b). These results demonstrated that miR-10a played important roles in regulating cell migration and invasiveness in GC and suggested that the down-regulation of miR-10a might contribute to tumor metastasis in gastric carcinogenesis.

**Figure 3:** miR-10a inhibits cell migration and invasion *in vitro*. **a** HGC-27 and MGC-803 cells were untreated or transfected with 50 nmol/L scramble or miR-10a for 24 h, and wounds were made. The relative ratio of wound closure per field is shown at 0, 12, 24, 36, 48 hours. Bar, 500 µm. **b** HGC-27 and MGC-803 cells were untreated or transfected with 50 nmol/L scramble or miR-10a for 24 h, and a transwell invasion assay was performed. The relative ratio of invasive cells per field is shown. Bar, 50 µm and 100 µm. All data are presented as the means ± SD. *, P<0.05; **, P<0.01, ***, P<0.001.

### miR-10a Targets HOXA1 in GC

MiRNAs perform biological functions through negatively regulating their target genes. It has been reported that the oncogene HOXA1 is a direct target of miR-10a in megakaryocytopoiesis and human pancreatic cancer [17]–[19]. As predicted by PicTar, there was a complementary sequence between has-miR-10a and HOXA1 3′UTR (FIG. 4a). However, it is unknown whether miR-10a regulates cell proliferation, migration and invasion in GC by targeting HOXA1. To clarify their regulatory relationship, we first detected the protein and mRNA levels of HOXA1 in miR-10a mimic-transfected HGC-27 and MGC-803 cells using western blotting and RT-PCR. We observed an evident decrease in the HOXA1 protein level in presence of miR-10a mimics compared with the scramble control in the two cells (FIG. 4b). The mRNA level of HOXA1 was also down-regulated in HGC-27 cells, suggesting that miR-10a inhibits HOXA1 expression by degrading mRNA of HOXA1 in HGC-27 cells. However, there was little alteration in the mRNA level of HOXA1 in MGC-803 cells, suggesting that miR-10a might down-regulate HOXA1 expression through translational repression but not mRNA cleavage in MGC-803 cells (FIG. 4c). Furthermore, we analyzed the protein levels of HOXA1 in 24 GC patients. Among these samples, there were 12 patients in whom miR-10a was down-regulated in their GC tissues and 12 patients in whom miR-10a was up-regulated in their GC tissues (FIG. 4d). HOXA1 was up-regulated in most of the patients in whom miR-10a was down-regulated in their GC tissues. Similarly, HOXA1 was down-regulated in most of the patients in whom miR-10a was up-regulated in their GC tissues. A comparison of miR-10a levels and protein levels of HOXA1 in GC revealed an inverse correlation between miR-10a and HOXA1 (r^2^ = 0.1839, P = 0.0366) (FIG. 4e). Collectively, these findings provide strong evidence that HOXA1 is a direct target of miR-10a in GC. We also detected the mRNA level of HOXA1 in these patients and observed that the mRNA level of HOXA1 in several patients was not consistent with the protein level which indicated that miR-10a regulates the expression of its target, HOXA1, through translational repression but not mRNA cleavage in these patients (FIG. S1).

**Figure 4:** miR-10a targets HOXA1 in GC. **a** The prediction of the binding between miR-10a and HOXA1 by Pictar. **b** HOXA1 protein expression in HGC-27 and MGC-803 cell transfected with miR-10a mimics. **c** HOXA1 mRNA level in HGC-27 and MGC-803 cell transfected with miR-10a mimics. **d** Western blot analysis of HOXA1 protein level in 24 GC patients. The left panel presents the expression of HOXA1 in 12 GC patients in whom miR-10a was down-regulated in their GC tissues (C) compared with the corresponding adjacent non-neoplastic tissues (N). The right panel presents the expression of HOXA1 in 12 GC patients in whom miR-10a was up-regulated in their GC tissues (C) compared to the non-neoplastic tissues (N). **e** Inverse correlation between HOXA1 protein levels and miR-10a expression in the above 24 GC patients.

### Knock-down of HOXA1 Suppressed Gastric Cancer Cell Growth and Migration *in vitro*

Next, we asked whether HOXA1 played important roles in gastric cancer cells. To examine the role of HOXA1 in GC, we knocked down endogenous HOXA1 in HGC-27 and MGC-803 cell lines to detect the effect on cell proliferation and cell migration. We observed that HOXA1 repression inhibited the cell proliferation and migration of HGC-27 and MGC-803 cells, respectively (FIG. 5a and 5b). These results suggest that miR-10a functions as tumor suppressor in GC cells by suppressing HOXA1 expression.

**Figure 5:** Knock-down of HOXA1 suppressed gastric cell growth and migration *in vitro*. **a** Growth assays by CCK-8 at 0, 1, 2, 3, 4 days after siHOXA1 transfection. **b** HGC-27 and MGC-803 cells were untreated or transfected with siHOXA1 or control for 24 h, and wounds were made. The relative ratio of wound closure per field is shown at 0, 12, 24, 36 hours. Bar, 500 µm. All data are presented as the means ± SD. *, P<0.05; **, P<0.01, ***, P<0.001.

### miR-10a is Epigenetically Silenced in GC Cell Lines

To elucidate whether the low expression of miR-10a in GC tissue was a result of epigenetical alterations, we treated HGC-27, MGC-803, SGC-7901 and MKN-45 cells with a DNA methylation inhibitor 5-AZA. The expression of miR-10a was up-regulated in HGC-27, SGC-7901 and MKN-45 cells when they were treated with AZA, suggesting that the expression of miR-10a might be repressed in these cells by DNA methylation (FIG. 6a).

**Figure 6:** miR-10a is epigenetically silenced in GC cell lines and GC patients. **a** Validation of the expression of miR-10a in HGC-27, MGC-803, SGC-7901 and MKN-45 cell lines treated with 5-AZA. **b** The genomic structure of *miR-10a* and its surrounding region. The CpG island is located at 1.6 kb upstream of *miR-10a*. Vertical ticks represent CpG sites. **c** qMSP analysis of the methylation level of the *miR-10a* genomic region in GC cell lines and after 5-AZA treatment. **d** The methylation level of the *miR-10a* genomic region in GC tissues (cancer) was higher than their matched adjacent non-neoplastic tissues (normal) in 55 GC patients. **e** The inverse correlation between miR-10a expression and the methylation status of the miR-10a genomic region in the investigated 55 GC patients. **f** The methylation level of the miR-10a genomic region in GES, HGC-27 and MGC-803 cells. All data are presented as the means ± SD. *, P<0.05; **, P<0.01, ***, P<0.001.

To study the regulation of miR-10a by DNA methylation, we searched the human genome database for the presence of CpG islands around miR-10a using “CpG Island Searcher” software and identified a CpG island located 1638 bp upstream of *miR-10a* (FIG. 6b). Further, we detected the DNA methylation status using qMSP and MSP in the four GC cell lines. The CpG island was hypermethylated in all four GC cell lines, which was consistent with the low expression of miR-10a in these GC cell lines. When the GC cells lines were treated with 5-aza-CdR, the methylation level was decreased compared with the DMSO group (FIG. 6c).

### The Down-regulation of miR-10a in GC Patients was due to the Hypermethylation of its CpG Islands

We further examined the methylation status of the CpG island in the GC tissue and the adjacent normal tissue of 55 randomly selected cases through qMSP. The methylation level in the 55 GC tissues was higher than that in the adjacent non-cancerous tissues (p<0.01), which was consistent with the low expression of miR-10a in GC tissues (FIG. 6d). In addition, we randomly selected two pairs of samples on which to analyze the DNA methylation level by bisulfate sequencing PCR (BSP) to validate the accuracy of MSP. The results of BSP were consistent with that of qMSP and were supplemented as FIG. S2. Furthermore, the methylation level of miR-10a (M/M+U) in these GC patients exhibited an inverse correlation with the expression of miR-10a (r^2^ = 0.1956, P = 0.0006) (FIG. 6e). We also detected the methylation level of miR-10a in normal gastric cells and gastric cancer cell lines. The results of qMSP revealed that the CpG island was partially methylated in GES cells but extremely hypermethylated in the two gastric cancer cell lines HGC-27 and MGC-803, which also suggested that the CpG island upstream of *miR-10a* was hypermethylated in GC cells (FIG. 6f). Collectively, these findings provide strong evidence that the expression of miR-10a was regulated by DNA methylation in these GC patients. The down-regulation of miR-10a in GC patients was due to the hypermethylation of its CpG islands.

## Discussion

In this study, we determined that miR-10a was down-regulated in human gastric cancer partially due to its DNA promoter hypermethylation. Further studies demonstrated that overexpression of miR-10a suppressed cell proliferation, migration and invasiveness in the GC cell lines HGC-27 and MGC-803, possibly through targeting the oncogene HOXA1.

MiRNAs have been reported to regulate various developmental and cellular processes, and are implicated in many human diseases, especially in cancer. MiRNAs suppress gene expression by targeting mRNAs through binding to their 3′ UTRs. These miRNAs exhibit regulatory roles in the pathogenesis of cancer and are involved in cell proliferation, differentiation, apoptosis, metastasis and resistance [4], [20]. MiR-10a plays an important role in several cancers, including hepatocellular cancer [9], pancreatic cancer [17], acute myeloid leukemia [21] and chronic myeloid leukemia [10]. The abnormal expression of miR-10a is likely to play a crucial role in malignant transformation and is relative to tissue-specificity. Its deregulation may contribute to the development of stomach neoplasia.

The validation of the expression of miR-10a in clinical samples demonstrated that miR-10a was down-regulated in 58 (58/100, 58%) GC tissues compared with the adjacent tissues. However, Weidong Chen *et al.* investigated the expression of miR-10a in 33 GC cases and observed that miR-10a expression was higher in GC tissues than in the adjacent tissues [22]. The inconsistency may be a result of the different quantity of clinical samples and the indistinctive change of miR-10a in GC tissues. Our data should be more biologically representive because of the larger numbers of clinical samples. Only a greater part but not all of the GC patients have a down-regulation of miR-10a in their GC tissues although miR-10a functions as a tumor suppressor in gastric cancer cells. This may be because of distinct mechanism of the genesis of GC in different individuals. There might be some other important genes or factors responsible for tumorigenesis in the GC patients in whose GC tissues miR-10a was unchanged or up-regulated. In addition, the miR-10a expression exhibited no correlation with clinicopathological characteristics except for TNM stage, indicating that miR-10a might play a partial role in tumorigenesis especially in early stages.

Many miRNAs have been reported to correlate with tumorigenesis, however, the underlying molecular mechanism remains unclear. In our report, a functional analysis of miR-10a, including cell proliferation, migration and invasion assays, helped us to better understand the contribution of miR-10a to gastric carcinogenesis. Transfection of miR-10a mimic significantly inhibited cell proliferation, migration and invasiveness in GC cells, indicating that the repression of miR-10a might promote tumor progression in gastric carcinogenesis. Future studies are needed to elucidate this mechanism.

In the human genome, *miR-10a* is located upstream of *HOXB4*. *MiR-10b*, another member of the miR-10 family, is located upstream of *HOXD4*. These two members are different from each other in only one base and exhibit identical seed sequences, suggesting their similar functions. Kwoneel Kim [12] has reported that miR-10b plays a role in GC as a tumor suppressor. In our study, we demonstrated that the overexpression of miR-10a inhibited tumor proliferation, migration and invasiveness, which was similar to the function of miR-10b in GC. HOX genes are highly conserved transcription factors that are determinant for correct anterior-posterior patterning of the body axis [23]. HOXA1 has been validated as a direct target of miR-10a in human pancreatic cancer [17] and megakaryocytopoiesis [18]. We also observed that the overexpression of miR-10a decreased HOXA1 protein levels in two GC cell lines, suggesting that HOXA1 is a direct target of miR-10a in gastric cancer.

Epigenetic modifications have been shown to be key mediators underlying the down-regulation of miRNA expression and exhibit a tight correlation with carcinogenesis [12], [13], [24]. Our data demonstrated that the hypermethylation of the CpG island upstream of *miR-10a* led to the down-regulation of miR-10a in GC cell lines and GC patients. Moreover, AZA treatment increased miR-10a in GC cell lines. Based on our findings, the methylation status of miR-10a may be employed as a potential biomarker in GC.

In summary, this study reports that miR-10a acts as a tumor suppressor in GC cells and is partly down-regulated by DNA hypermethylation. Forced expression of miR-10a suppresses cell proliferation, migration and invasiveness *in vitro*. The methylation status and the expression level of miR-10a may serve as potential biomarkers of GC, and miR-10a may have potential therapeutic value in cancer therapy. Further studies on the epigenetic regulation of miRNA expression are necessary, and the regulation of miRNA expression by epigenetic drugs may provide a novel therapeutic strategy for gastric and other human cancers.

## Supporting Information

Figure S1 The mRNA level of HOXA1 in the 24 GC patients was detected by qRT-PCR.
(TIF)

Figure S2 BSP analysis of the methylation status in two GC patients. Filled and open circles represent methylated and unmethylated CpG sites respectively.
(TIF)

Table S1 The primers are used in this article.
(XLSX)

Table S2 Association between the expression of miR-10a with clinicopathological features in patients with gastric cancer.
(XLSX)
